# A Network Pharmacology-Based Study on Irritable Bowel Syndrome Prevention and Treatment Utilizing Shenling Baizhu Powder

**DOI:** 10.1155/2021/4579850

**Published:** 2021-11-23

**Authors:** Meng Meng, Chen Bai, Bo Wan, Luqing Zhao, Zhe Li, Danyan Li, Shengsheng Zhang

**Affiliations:** ^1^Digestion Center, Beijing Hospital of Traditional Chinese Medicine, Capital Medical University, Beijing, China; ^2^Beijing University of Chinese Medicine, Beijing, China; ^3^Center for Stem Cells and Regenerative Medicine, King's College London, Guy's Hospital, Great Maze Pond, London, UK

## Abstract

**Methods:**

Metabolomics was used to detect the secondary metabolites in SLBZP; the target protein was acquired by target fishing according to the compound's structure. The SymMap database was used to search herbal medicines for the target protein. The target gene of IBS gave rise to the common gene protein which is the potential target of SLBZP in IBS therapy. The interactions between target proteins were analyzed in a STRING database, the protein relationship network was analyzed using Cytoscape software, and the Kyoto Encyclopedia of Genes and Genomes enrichment analysis of the core target gene group was carried out in a DAVID database in order to construct the “compound-traditional Chinese medicine/molecule-target-pathway” network. Molecular docking was used to verify the core protein and its related small molecular compounds.

**Result:**

There were 129 types of secondary metabolites in SLBZP. 80 target proteins of these metabolites were potential core targets for IBS treatment including acetylcholinesterase (AChE), arachidonate-5-lipoxygenase (ALOX5), B-cell lymphoma-2 (BCL2), recombinant cyclin D1 (CCND1), and catenin-*β*1 (CTNNB1), among others. Results from these targets indicated that the most enriched pathway was the tumor necrosis factor (TNF) signaling pathway (*p* < 0.001) and that the most abundant pathway was signal transduction. In the network nodes of the TNF signaling pathway, the Chinese medicines with the highest aggregation were Lablab semen album and Glycyrrhizae radix et rhizoma (degree = 11). The small molecules with the highest aggregation were oxypeucedanin and 3,5,6,7,8,3′,4′-heptamethoxyflavone (degree = 4). Molecular docking results confirmed that daidzein 7-O-glucoside (daidzin) had the highest degree of binding to TNF proteins in the TNF signaling pathway.

**Conclusion:**

This study shows that SLBZP can treat IBS by influencing multiple targets and pathways, of which the TNF signaling pathway may be the most significant. This typifies the pharmacological characteristics of traditional Chinese medicine, i.e., multiple targets, numerous pathways, and specific therapeutic effects on diseases. SLBZP can therefore be used as a candidate drug for clinical IBS by intervening in human signal transduction.

## 1. Background

Irritable bowel syndrome (IBS) is one of the most frequently arising pathologies of the gastrointestinal tract presenting in the clinic. Its main manifestations are pain and discomfort within the abdomen, together with changes in bowel habits. With an incidence rate range of 7% in Southeast Asia to 21% in South America [1], IBS affects hundreds of millions of people. The pathogenic factors include alterations in the microbiome, permeability, peristalsis, and immune function of the intestine, as well as changes in the brain-gut axis and social psychological status, among others [2]. IBS is divided into four subtypes according to defecation habits: (i) constipation (IBS-C); (ii) diarrhea (IBS-D); (iii) mixed (IBS-M); and (iv) undetermined (IBS-U). The first-line treatment of IBS usually includes exercise and diet control, fiber supplements, probiotics, antispasmodics, and secretagogues [3]. Although IBS is a prevalent complaint and these drugs target specific symptoms, they have little effect on systemic symptomatology or abdominal pain and distension [4].

Shenling Baizhu powder (SLBZP) is derived from the “Prescriptions of Taiping Heji Bureau” (1148 A.D.) in the Song Dynasty of China. Its constituents include white lentils, Atractylodes macrocephala, Poria cocos, licorice, Platycodon grandiflorum, lotus seed, ginseng, Amomum villosum, yam, and coix seed. The main clinical effects of the drug are splenic and gastric fortification and replenishment and restoration of lung qi. In China, it is principally used to alleviate clinical symptoms such as splenic and gastric inadequacy, anorexia, loose motions, shortness of breath, cough, and limb fatigue. To date, several pharmacological studies have been published relating to SLBZP, as shown in Table 1, suggesting that it can exert therapeutic effects on several gastrointestinal diseases via a spectrum of pharmacological approaches [5–13]. A systematic review of studies evaluating the treatment of IBS with SLBZP indicated that the mixture was safe and effective in enhancing the cure rate of IBS and diminishing the severity of diarrhea, abdominal pain, and distension [14]. However, there is little research relating to its mechanism of action in such patients.

In 2007, Hopkins, from the United Kingdom, proposed the concept of network pharmacology which takes the biological databases as the processing object [15]. From the perspective of systems biology, using an empirical interaction network of pathologies, phenotypes, genomes, targets, and pharmaceutical agents, network pharmacology facilitates the observation of the intervention and influence of drugs on the pathological network. This is achieved through network topology, target criterion, and classification analyses, respectively, together with other computational analytical methods, enabling drug research and development protocols to resemble actual pathological scenarios more closely. Network pharmacology systematically understands the dynamic changes of human diseases and the interaction of multiple factors in the pathophysiological process. This is highly consistent with the characteristics of the numerous drug components and corresponding multiple targets of compounds utilized in traditional Chinese medicine.

A network pharmacology method was deployed in the current research in order to construct the “compound-traditional Chinese medicine/molecule-target-pathway” network of SLBZP for the treatment of IBS and to explore its potential pharmacological mechanism. The flow chart of the entire research design is shown in Figure 1. The potential targets of SLBZP with respect to IBS therapy were acquired using metabolomics technology, target fishing, and database matching methods. The core targets were enriched and analyzed, and then the “compound-traditional Chinese medicine/molecule-target-pathway” network was configured. The results obtained during this work will offer a data reference for the research and development of de novo drugs for other treatable diseases and IBS with respect to SLBZP.

## 2. Results

### 2.1. Compound Secondary Metabolites

As shown in Figure 2, a total of 129 secondary metabolites were recognized within the compound granules, which were sorted in descending order according to the integrated area of mass to charge ratio mass spectrometry response. The top five percent were as follows: bis(N,N-diethylethanaminium)-2-acetamido-1,5-anhydro-2-deoxy-1-[-hydroxy(phosphonato)methyl]-D-glucitol (relative content 6.49 × 10^7^); glycyroside (relative content 4.81 × 10^7^); apigenin 6,8-C-diglucoside (relative content 4.20 × 10^7^); acacetin-7-O-glucuronide (relative content 4.00 × 10^7^); and trigonelline (relative content 3.88 × 10^7^). Fifty-eight types of flavonoids were noted, of which the following 21 were most abundant (as shown in Figure 3): apigenin 6,8-C-diglucoside; acacetin-7-O-glucuronide; licoflavone C; acacetin-7-O-galactoside; luteolin-7-O-rutinoside; isosinensetin; luteolin-6,8-di-C-glucoside; diosmin; luteolin-7-O-glucoside (cynaroside); nobiletin; baicalin; luteolin-7-O-glucuronide; diosmetin-7-O-galactoside; 5-hydroxy-6,7,8,3′,4′-pentamethoxyflavone; 8-methoxychrysin (wogonin); tetramethyl-O-isoscutellarein; diosmetin-7-O-glucuronide; isorhamnetin-3-O-rutinoside (Narcissin); Sudachiin B; apigenin; and apigenin O-hexosyl-O-pentoside.

### 2.2. Targets of SLBZP in the Treatment of IBS

As shown in Figure 4, a total of 1073 secondary metabolite-related targets, 618 targets included in the database, and 456 IBS-related targets were obtained. Among them, 80 target proteins were shared proteins, which were the target genes related to the treatment of IBS by SLBZP, as shown in Table 2.

### 2.3. Target Interaction Network

As shown in the results of the target interaction network in Figure 5, there were 1023 intertarget relationships among 80 targets; on average, each target had potential interactions with 26 targets. The local clustering coefficient was 0.662, and the protein-protein interaction (PPI) enrichment *p* value was <0.001, suggesting that as a cohort, the proteins were biologically connected to some extent. A total of 5 subnetworks were obtained following cluster analysis of this network, as shown in Figure 6. Among them, cluster 1 had the highest cluster score; this subnetwork contained 30 target proteins, as shown in Table 2. These proteins were the core targets of SLBZP in IBS therapy.

### 2.4. The Results of Pathway Cluster Analysis

As shown in Figures 7–9, a total of 89 pathways were obtained from the enrichment of core target groups, including 4 categories and 17 subcategories in the Kyoto Encyclopedia of Genes and Genomes (KEGG) database. The four first-level classification categories and proportions among them were human diseases (49.4%), organismal systems (28.1%), environmental information processing (19.1%), and cellular processes (3.4%). The pathway with the highest degree of enrichment was the tumor necrosis factor (TNF) signaling pathway (*p* < 0.001); the most abundant pathway was signal transduction.

### 2.5. The Results of Pathway Enrichment Analysis

Figures 10 and 11 display the constructed first-level classification pathways of non-“human diseases” and the network with related targets and Chinese medicines. In the total network nodes, Lablab semen album (degree = 29), transferulic acid (degree = 12), and TNF signaling (degree = 14) were the most aggregated traditional Chinese medicine, small molecule, and pathway, respectively. In the network nodes of the TNF signaling pathway, the Chinese medicines with the highest aggregation were Lablab semen album and Glycyrrhizae radix et rhizoma (degree = 11), and the small molecules with the highest aggregation were oxypeucedanin and 3,5,6,7,8,3′,4′-heptamethoxyflavone (degree = 4).

### 2.6. The Results of Molecular Docking

According to the above results, molecular docking of the TNF protein was carried out; the results are shown in Figure 12. Daidzein 7-O-glucoside (daidzin) was the most closely bound to TNF with a binding energy of -10.3 kcal/mol; it interacted with 11 amino acids by hydrogen bonds.

## 3. Discussion

There are many causes of IBS, but the etiology is still not clear. Studies have shown that IBS may occur following only slight changes and disturbances, such as the improvement of modern social health conditions or personal hygiene habits or short-term infection or stress [16]. Owing to the complexity of the causes of the disease, there is a wide selection of potential treatments. IBS can seriously affect patients' quality of life and occupational productivity [17]. The total cost of IBS treatment in China has reached 123.83 billion yuan.

In 2018, the American Society of Gastroenterology published a consensus opinion on IBS therapy [3], recommending that in addition to nondrug therapies such as exercise and diet control, secretagogues such as linaclotide and plecanatide and cellulose drugs should be offered for IBS-C. Eluxadoline and alosetron are suggested for IBS-D, but the quality of evidence for this is weak. However, each treatment has its own indications and contraindications, together with inevitable adverse event profiles. For example, linaclotide is generally considered to be a safe and well-tolerated drug, but dose-dependent diarrhea still occurs [18]. In addition, the http://Drugs.com/ database suggests that in nonclinical studies on newborn mice, a single oral dose of linaclotide can cause dehydration and death, as well as abdominal pain, stomach ache, severe diarrhea, and other common side effects. Eluxadoline increased the risk of pancreatitis. In the United States, adverse event logs relating to eluxadoline, recorded between January and September 2016, revealed that 98 patients with IBS-D had pancreatitis due to taking eluxadoline, resulting in 2 deaths [19]. It is therefore paramount to discover an efficacious, safe, and cost-effective drug which could even be used for the early clinical issues that arise before IBS becomes a major priority.

There are ten kinds of Chinese herbal medicine in SLBZP, among which lentil is the sovereign medicine. Studies have suggested that lentils within this compound are a potential core Chinese workhorse. The traditional Chinese medicine, white lentil, is the dried mature seed of the legume lentil Dolichos lablab L., which was first recorded in the “famous doctors' records” in the late Han Dynasty over 1500 years ago. In the *Chinese Pharmacopoeia 2015 Edition*, it is documented that this substance can be used as therapy for IBS-related clinical symptomatology, such as loss of appetite, loose stools, and abdominal discomfort, as shown in Figure 13. Among the detected secondary metabolites, most of them have been proven to have certain anti-inflammatory, systemic, and regeneration-promoting effects, of which oxypeucedanin and 3,5,6,7,8,3′,4′-heptamethoxyflavone were deemed the most enriched. Oxypeucedanin is an open channel blocker, acting on the hKv1.5 channel [20], and can inhibit the growth and cellular life cycle of melanoma cells [21]. Heptamethoxyflavone substances can participate in the regulation of platelet antiadhesion activity [22]. Lentil is the homologous product of medicine and food. It has no toxic side effects on the human body after reasonable cooking, while oxypeucedanin and 3,5,6,7,8,3′,4′-heptamethoxyflavone are small molecular compounds with certain potential pharmacological properties, so they can be used as possible follow-up research and development drugs.

Among the disease pathways suggested by the KEGG database pathway enrichment results, in addition to tuberculosis, pertussis, and other pathology pathways that are not directly related to IBS, there are predominantly two kinds of IBS-related diseases, i.e., inflammatory bowel disease (IBD) and colorectal cancer. IBS and IBD are two completely different pathologies. At present, with respect to the relationship between the two, studies have pointed out that about one-third of patients with IBD have persistent intestinal sensation and movement and intestinal flora abnormalities, which may cause symptoms similar to IBS [23]. In terms of the relationship between IBS and colorectal cancer, some studies have suggested that no association between these disease processes has been found. However, it is clear that there are many cases of misdiagnosis caused by similar symptoms [24]. Combined with the results of this study, in addition to IBS, SLBZP may also be used as a potential candidate drug for IBD and colorectal cancer.

TNF was selected for molecular docking because as an important cytokine, it is able to trigger a variety of intracellular signal pathways and is the initiating factor of the TNF signal pathway. Activated TNF will activate this pathway and induce downstream leukocyte recruitment and inflammatory factor release. It is involved in inducing cellular necrosis and survival, inflammation, and immunity. One of the most significant proinflammatory cytokines, TNF-*α*, is a principal factor in vasodilation and edema and in the epithelial adhesion of leukocytes through adhesion molecule expression. It also governs hemostasis, promotes oxidative stress in inflammatory areas, and indirectly gives rise to pyrexia [25]. At present, studies have suggested that there is an imbalance of TNF in patients with IBS [26]. This change may be related to the release of intestinal microbiota and brain neurotransmitters, mediated via the “brain-gut-bacteria” axis [27]. Although IBS is not an inflammatory disease per se, it is undeniable that its pathological features have similar inflammatory manifestations. Early inhibition of an inflammatory response through anti-inflammatory agents may therefore be an effective IBS treatment. Such substances include daidzin in SLBZP, which has been shown to offer a certain degree of anti-inflammatory influence through the TNF signaling pathway [28]. Thus, it is concluded that the latter is the mechanism through which SLBZP mainly exhibits an anti-inflammatory effect.

## 4. Conclusion

To summarize, a network, founded on network pharmacology technology, was constructed in order to predict the interaction between substances in SLBZP and target genes. The data demonstrated that SLBZP may be a significant factor in IBS therapy by acting on the TNF signaling pathway. Based on the analysis of systems biology, it was speculated that SLBZP may not only be a player in multiple mechanisms that combine synergistically to treat IBS but also contribute to factors that diminish the IBS incidence. In addition, SLBZP may also be a potential treatment for IBD and colorectal cancer. However, the results obtained by systems biology analysis still need to be verified by pharmacological methods with the aid of omics technology.

## 5. Method

### 5.1. Metabolomics Analysis

#### 5.1.1. Sample Preparation and Extraction

Three sachets, each containing 6 g of SLBZP (Beijing Tongrentang Pharmaceutical Co., Ltd.), were used for the study (in order to ensure the stability of the results, one bag was used for each measurement, and the measurement was repeated 3 times). The substance was comminuted for 90 seconds in a mixer mill (MM 400, Retsch) with zirconia beads at 30 Hz. Centrifugation was then performed at 10,000 g for a period of 10 minutes. The extract was absorbed (CNWBOND Carbon-GCB SPE Cartridge, 250 mg, 3 mL; ANPEL, Shanghai, China). Filtration was then performed prior to analysis by liquid chromatography-electrospray ionization-mass spectrometry (LC-ESI-MS).

#### 5.1.2. High-Performance Liquid Chromatography Conditions

An LC-ESI-MS system (high-performance liquid chromatography (HPLC) and Shim-pack ultraperformance liquid chromatography (UFLC), Shimadzu CBM30A system; mass spectrometry (MS), Applied Biosystems 6500 triple quadrupole-linear ion trap (QTRAP)) was used to analyze the resulting extracts. The following analytical conditions were employed: HPLC column: Waters ACQUITY UPLC HSS T3 C18 (1.8 *μ*m, 2.1 mm∗100 mm); solvent system: water (0.04% acetic acid) and acetonitrile (0.04% acetic acid); and gradient program: 100 : 0 *V*/*V* at 0 min, 5 : 95 *V*/*V* at 11.0 min, 5 : 95 *V*/*V* at 12.0 min, 95 : 5 *V*/*V* at 12.1 min, and 95 : 5 *V*/*V* at 15.0 min. A flow rate of 0.40 mL/min was utilized; the temperature was maintained at 40°C, and 2 *μ*L injection volume was used. The effluent was alternately connected to an electrospray ionization-triple quadrupole-linear ion trap-mass spectrometry (ESI-QTRAP-MS/MS).

#### 5.1.3. ESI-QTRAP-MS/MS

The linear ion trap (LIT) and triple quadrupole (QQQ) scans were acquired on a QQQ-LIT (QTRAP) mass spectrometer and an API 6500 QTRAP LC/MS/MS system. The system incorporated an electrospray ionization (ESI) turbo ion spray interface, which operated under positive ion mode, and was controlled by Analyst 1.6.3 software (AB Sciex). The following working parameters of the ESI source were deployed: ion source and turbo spray; source temperature 500°C; ion spray voltage 5500 V; and ion source gas I and gas II and curtain gas at 55, 60, and 25.0 psi, respectively; collision gas was high. The instrument was tuned and mass calibrated with 10 *μ*mol/L and 100 *μ*mol/L propylene glycol solutions in QQQ and LIT modes, respectively. The QQQ scans were obtained as multiple reaction monitoring (MRM) experiments; collision gas (nitrogen) was set to 5 psi. The declustering potential and collision energy of a single MRM conversion were further optimized. In accordance with the metabolites eluted during this period, a specific set of MRM transitions was monitored for each timeframe.

#### 5.1.4. Qualitative Analysis of Metabolites

Based on the Malware Database (MetWare) and public databases of metabolite information, respectively, the primary and secondary MS spectrum data were analyzed qualitatively. Iterative isotope signals containing potassium, sodium, and ammonium ions, together with repeating signals of fragment ions of other high-molecular weight compounds, were removed in the process. The structure of metabolites was analyzed with reference to MassBank, KNAPSAcK, the Human Metabolome Database (HMDB) [29], the Metabolome Tomato Database (MoTo DB), and the Metabolite Link (METLIN) [30] as well as to additional existing mass spectrometry public databases.

### 5.2. Network Pharmacology Analysis

#### 5.2.1. Prediction of Potential Targets of SLBZP in the Treatment of IBS

Searches were performed in PubChem and ChemSpider databases to determine the molecular structure of small compounds obtained by metabolomics. The database SwissTargetPrediction was utilized for target fishing in order to obtain related targets for secondary metabolites. The SymMap database was utilized to search for all known target proteins of traditional Chinese medicines within SLBZP [31]; these were merged with the medicine targets. Duplicates were eradicated so as to retain the unique values. A search for IBS genes was conducted using the Comparative Toxicogenomics Database. Retaining the secondary metabolite targets, the known targets in the database and the common gene targets of IBS genes produced the potential targets of SLBZP in IBS treatment.

#### 5.2.2. Constructing a Network of Interaction Relationships between Analytical Targets

The potential targets of the proven prescriptions for the treatment of diarrhea were entered into the STRING database, the organization selected was “Homo sapiens,” and the function “search” was clicked in order to analyze and obtain the PPI. The PPI network was imported into Cytoscape (v3.7.2) software, and the MCODE plugin was used to cluster the PPI network in order to obtain the core target group for the treatment of diarrhea.

#### 5.2.3. Construction of the Core “Molecule-Target-Pathway” Network

The core target group was entered into the DAVID database in order to perform enrichment analysis and to obtain the potential KEGG pathway. In the acquired pathways and according to the relationship between a target and the corresponding Chinese medicine, Cytoscape (v3.7.2) software was utilized in order to build a “Chinese medicine-molecule-target-pathway” network of nonspecific disease pathways so as to visualize the network relationship.

#### 5.2.4. Molecular Docking Analysis

Molecular docking was used to verify the marker proteins in the most enriched pathway. The 3-dimensional structure of the human target protein was downloaded from the Protein Data Bank (PDB) with the PDB ID of “1TNF” and stored in PDB format. Dehydration and hydrotreatment of the protein were carried out using AutoDockTools (v4.2) software and saved in PDBQT format. Following energy minimization, the 3-dimensional structure of the small molecular compound relating to SLBZP was saved in PDBQT format. The structure of the small molecule and the corresponding target protein was imported into PyRx (v0.9.8) software, and the AutoDock Vina algorithm was employed for molecular docking. According to the docking scoring results, the combination potential between the two was evaluated. The docking results were exported as PDB files; PDB format files of ligand-receptor binding were generated by PyMOL (v2.4.1) software, and 2-dimensional structure diagrams of ligand-receptor binding were generated by LigPlot (v4.5.3) software.

## Figures and Tables

**Figure 1:** Research design flow chart.

**Figure 2:** Qualitative and quantitative detection results of secondary metabolites in compound granules. Note that (a) shows the total ion flow diagram of mass spectrometry analysis of mixed samples and (b) shows the multipeak diagram of MRM metabolite detection. Left: positive ion current; right: negative ion current.

**Figure 3:** Primary and secondary classifications of secondary metabolites. Note that the number is the number of detection times. The inner and outer circles are the first- and second-level classifications, respectively.

**Figure 4:** Venn diagram of target genes related to IBS treated with SLBZP.

**Figure 5:** Intertarget interaction network of SLBZP in the treatment of IBS.

**Figure 6:** Cluster analysis results of the target interaction network of SLBZP in the treatment of IBS. Note that the warmer the node color, the higher the importance of the node in the network.

**Figure 7:** Core target pathway enrichment bubble chart of SLBZP in IBS therapy (top 25%).

**Figure 8:** Double-loop diagram of enrichment and classification of the core target pathway of SLBZP in IBS therapy.

**Figure 9:** Enrichment results of the TNF signaling pathway. Note that the red pentagram is the protein mapped from SLBZP.

**Figure 10:** The “drug-molecule-target-pathway” network of SLBZP in the treatment of IBS. Note that the green diamond node is the traditional Chinese medicine, the green arrow node is the molecule, the circular node is the target protein, the hexagonal node is the pathway, and the three parts from top to bottom represent cellular processes, environmental information processing, and organic systems, respectively. The yellow node is the TNF signaling pathway and its related proteins.

**Figure 11:** The “drug-molecule-target-pathway” network of SLBZP in treating IBS through the TNF signaling pathway. Note that the green diamond node is the traditional Chinese medicine, the green arrow node is the molecule, the circular node is the target protein, and the hexagonal node is the pathway. The yellow nodes are TNF proteins, related small molecules, and traditional Chinese medicine.

**Figure 12:** Docking results of TNF-related molecules and their binding energies: (a) eucommiol, -6.2 kcal/mol; (b) calycosin, -8.9 kcal/mol; (c) N-p-coumaroyl-N′-feruloylputrescine, -7.4 kcal/mol; (d) 49.N-*cis*-feruloyltyramine, -8.6 kcal/mol; (e) daidzein-4′-glucoside, -8.0 kcal/mol; (f) 79.formononetin 7-O-*β*-D-glycoside, -10.4 kcal/mol; (g) daidzein 7-O-glucoside (daidzin), -10.3 kcal/mol; (h) genistein 8-C-glucoside, -9.4 kcal/mol.

**Figure 13:** Lentil-related “molecule-target-disease-symptom” relationship network. Note that data is from the SymMap database.

**Table 1:** Research overview of studies relating to SLBZP in the treatment of digestive system diseases, listed in descending order of publication year.

Article	Disease	Research	Position of action mechanism
Chao et al. [5]	Ulcerative colitis	Mice	The MAPK/NF-*κ*B and pyroptosis signaling pathway
Ji et al. [6]	Chronic diarrhea	Rats	Intestinal absorption function and mucosal ultrastructure
Zhang et al. [7]	Functional dyspepsia	Rats	Intestinal microbiota
Lv et al. [8]	Inflammatory bowel disease	Rats	Intestinal microbiota
Shi et al. [9]	Diarrhea	Rats	Intestinal microbiota
Lv et al. [10]	Antibiotic-associated diarrhea	Rats	Intestinal microbiota
Son et al. [11]	Cancer of the liver	Mice	Tumor growth promoter, antiapoptotic protein, and proapoptotic protein
Yang et al. [12]	Nonalcoholic fatty liver disease	Rat Kupffer cells	p38 MAPK pathway
Chao et al. [13]	Colon cancer	Human	Ghrelin

**Table 2:** SLBZP for the treatment of IBS-related target genes. Bold italics are the core targets.

***CCND1***	***CASP3***	***MMP9***	ACHE	PGR	HTR3A	XIAP	PLA2G4A
***IL1B***	***GAPDH***	***MPO***	ALOX5	PLA2G2A	NQO1	GCG	CCR2
***JUN***	***HMOX1***	***RELA***	BCL2	PON1	OPRD1	APP	NR1H3
***NOS2***	***ICAM1***	***SELE***	CTNNB1	PTGS1	OPRK1	CASP7	GABBR1
***NR3C1***	***IL2***	***STAT1***	ESR1	CYP1A1	PARP1	PTGES	RXRA
***PPARG***	***MAPK1***	***VCAM1***	GSK3B	CYP1A2	PPARA	GLA	SLC6A2
***PTGS2***	***MAPK3***	***MAPK8***	KCNH2	CYP3A4	RXRB	MMP13	SLC6A3
***TNF***	***MMP1***	***ELANE***	MAOA	DRD2	SELP	MMP7	SLC6A4
***VEGFA***	***MMP2***	***STAT3***	MAOB	GSR	TH	RPS6KB1	XDH
***AKT1***	***MMP3***	***TLR4***	OPRM1	GUSB	TRPV1	CYP2D6	ABCB1

## Data Availability

All data are available in the manuscript, and they are shown in figures, tables, and supplementary files.

## Abbreviations

IBS: Irritable bowel syndrome
SLBZP: Shenling Baizhu powder
AChE: Acetylcholinesterase
ALOX5: Arachidonate-5-lipoxygenase
BCL2: B-cell lymphoma-2
CCND1: Recombinant cyclin D1
CTNNB1: Catenin-*β*1
TNF: Tumor necrosis factor
IBS-C: Irritable bowel syndrome-constipation
IBS-D: Irritable bowel syndrome-diarrhea
IBS-M: Irritable bowel syndrome-mixed
IBS-U: Irritable bowel syndrome-undetermined
PPI: Protein-protein interaction
KEGG: Kyoto Encyclopedia of Genes and Genomes
IBD: Inflammatory bowel disease
LC-ESI-MS: Liquid chromatography-electrospray ionization-mass spectrometry
HPLC: High-performance liquid chromatography
UFLC: Ultraperformance liquid chromatography
MS: Mass spectrometry
QTRAP: Triple quadrupole-linear ion trap
ESI-QTRAP-MS/MS: Electrospray ionization-triple quadrupole-linear ion trap-mass spectrometry
LIT: Linear ion trap
QQQ: Triple quadrupole
ESI: Electrospray ionization
MRM: Multiple reaction monitoring
HMDB: Human Metabolome Database
MoTo DB: Metabolome Tomato Database
METLIN: Metabolite Link
PDB: Protein Data Bank.

## Supplementary Materials

Supplementary Materials Please find detailed data in the supplementary file, including the original data of SymMap, metabolomics, and molecular docking of Shenling Baizhu powder. “Shenling Baizhu powder SymMap” includes all herbal targets and combined targets. “Shenling Baizhu powder metabolomics” includes two-dimensional structural data analysis. “Molecular docking” involves molecule-target docking and the results.
